This article has been retracted.

# Application of Free Skin Flap Transplantation in Skin Malignant Tumor Resection

**DOI:** 10.1155/2022/7510330

**Published:** 2022-04-18

**Authors:** Yue Zhou, Weili Xu, Jue Hou, Chunsheng Hou, Jufang Zhang

**Affiliations:** ^1^Nanjing Medical University, Nanjing, Jiangsu, China; ^2^Zhejiang Chinese Medical University, Hangzhou, Zhejiang, China; ^3^Affiliated Hangzhou First People's Hospital, Zhejiang University School of Medicine, Hangzhou, Zhejiang, China; ^4^The Affiliated Hangzhou Hospital of Nanjing Medical University, Nanjing, Zhejiang, China

## Abstract

One of the most important surgical approaches for restoring cutaneous abnormalities caused by tumor resection is the insertion of a skin flap. Flap transplantation has been used to cover and fill different deficiencies after tumor removal. However, distal necrosis is among the most prevalent postsurgical consequences for skin flaps, particularly when treating large regions. Blood circulation failure causes flap necrosis, which may lead to serious problems, particularly in patients undergoing body cavity reconstruction following tumor excision. ADSCs (adipose-derived stem cells) are a kind of stem cell separated from the adipose tissue that has multilineage differentiation, simple availability, high proliferation capability, and self-renewal capabilities. This paper uses human adipose-derived stem cell (ADSC) therapy for skin flap transplantation in skin malignant tumor resection. ADSC-based therapy is an applicable technique for assisting flap transplantation. The isolation of ADSC is performed using different trypsin concentrations, and then, the population doubling time is determined. The isolated ADSCs are differentiated and then employed for the skin flap model. The performance of the suggested method is analyzed using various assays. The usage of adipose-derived stem cells to boost the vitality of the skin flaps proved successful.

## 1. Introduction

Current data study has indicated that skin malignant tumors are common, with basal cell carcinomas and squamous cell carcinomas responsible for the majority of cases (approximately 65 percent). Surgical resection is the most common therapeutic procedure for tumors, particularly cancerous tumors. One of the most frequent injuries in skin tumor surgical resection is skin malformation. The majority of wound infections are open wounds with skin abnormalities. Skin flaws are present in more than half of all acute wounds. Direct stitches, skin transplantation, local skin flap transference repair, remote skin flap transplantations, free skin flap transplantations, skin tissue expansion restoration, and other techniques are routinely employed in medical therapy to repair wound abnormalities. Facial plastic surgery is the oldest utilization of skin flaps. Skin flap treatment ushers in wonderful developments with the development of microsurgery. One of the most efficient ways for repairing large-area skin and soft tissue abnormalities as well as surgical scar rigidity is free skin flap transplantation [1–5].

The desire to substitute or rejuvenate injured cells is increasing as a result of age-related and other degenerative disorders, malignancies, wounds, and congenital defects. To restore injured cells, the very first phase of regenerative therapy is using differentiated cells obtained through biopsies, cultivated in vitro and transplanted onto appropriate substrates made of synthetic and/or organic substances. Differentiated cells have the phenotypic characteristics required for a specific purpose and perform desired biological functions like creating an ordered extracellular matrix (ECM), secreting certain signaling molecules, and communicating appropriately with adjacent cellular membranes. Yet, the tiny handful of harvested cells and its weak multiplication ability while grown in vitro limit the utilization of differentiated cells in tissue regeneration. It is particularly true for the aged and polymorbid, who require regeneration therapies. Regardless of the fact that some organs, such as the liver, have a high propensity to regenerate in vivo, and growing and multiplying cells from such organs in vitro may be problematic [2, 6, 7].

Despite significant advances, major full-thickness skin defects continue to be linked with death because of a scarcity of donor skin locations. Autologous CEAs (cultured epidermal autografts) were the first epidermal substitutes, but their functional and aesthetic outcomes were unsatisfactory owing to graft contracture, scarring, and infections. New cell sources have been utilized for skin tissue regeneration due to a scarcity of skin donor sites after major full-thickness skin injuries. Adult stem cells from adipose tissue are numerous and easy to obtain for translational therapeutic techniques such as skin tissue engineering [3, 4, 8–10]. Several authors have illustrated various methodologies over skin flap transplantation in skin malignant tumor resection [11]. In order to identify whether the approach was preferable than the other in line with current European and US regulations, researchers examined two ways of adipose-derived stem cell (ADSC) extraction, one based on a mechanical + enzymatic (ME) process and the other just mechanical (MC). According to the data acquired, the ME approach was able to isolate a larger number of ADSCs (25.9%) from the same quantity of lipoaspirate as the MC procedure (5%) [12]. In order to give thorough knowledge regarding the threefold role of exosomes in transplantation therapy, we attempted to compile a list of resources. Palumbo et al. [13] summarized the literary works and offer a comprehensive summary of the methodological challenges concerning human ADSC separation, preparation, characterization, growth, and differentiation methods, remembering their core concepts, benefits, and constraints while focusing on how these processes may impact ADSC performance, functionality, and plasticity. Hu et al. [14] examined the impact of adipose-derived stem cell-derived exosomes (ADSC-Exos) on angiogenesis following skin flap transplantation in rats. By increasing neovascularization following skin flap transplantation, ADSC-Exos can enhance the blood supply of skin flaps and thereby increase the survival rate of skin flaps in rats. Pu et al. [15] investigated if ADSCs and their derivatives may promote neovascularization and preserve skin flaps following I/R damage. The direct development of ADSCs into endothelial cells and the indirect action of IL-6 generated by ADSCs are both parts of the skin healing process. Off-the-shelf medicines such as ADSC-CM and ADSC-Exo might be utilized for this treatment. Bai et al. [16] investigated if exosomes produced from ADSC can preserve the skin flap and stimulate neovascularization following ischemia-reperfusion (I/R) damage. In [17], Yadav and Shrestha examined the most popular microvascular free flaps (MFF) utilized in OMF reconstruction, including the radial forearm free flap (RFFF), anterolateral thigh flap (ALT), and free fibula flap (FFF). They are rightly referred to as the workhorses of OMF reconstruction in terms of free flaps since they can accommodate practically all large abnormalities we see following ablative surgery in the OMF region. In [18], Mohamed-Ahmed et al. investigated the multiplication, differentiation capacity, and probable impacts of donor variability on donor-matched adipose-derived stem cells (ADSCs) and bone marrow mesenchymal stem cells (BMSCs). In [19], Si et al. summarized the present landscape of ADSC isolation, identification, localization, and differentiation ability as well as recent advancements in ADSC applications, the newest preclinical and clinical research, and future approaches for the use of ADSCs. In [20], Megaloikonomos et al. discussed all significant aspects for ADSC cultivation, culture, distinction, and phenotypic categorization, offering a holistic framework of such a procedure, classifying the distinctions between ADSCs gathered from multiple rat adipose tissues and offering FT-IR spectroscopy indicator bands, which could be used as fingerprints to distinguish the categories of adipose tissues.

Hence, in this paper, human adipose-derived stem cell (ADSC) therapy is used for efficient skin flap transplantation in skin malignant tumor resection. The further parts of the paper are organized as follows: Section 2 explains the problem statement.  Section 3 explains the suggested methodology.  Section 4 analyzes the behavior of the suggested method. Also, finally, Section 5 concludes the overall idea of the paper.

## 2. Problem Statement

Both embryonic stem cells and induced pluripotent stem cells have theoretical advantages, but they also have certain disadvantages. Adult stem cells, on the other hand, are more widely available, and as long as they are produced from autologous tissue, there are no ethical or immunological problems. Adipogenic, osteogenic, chondrogenic, myogenic, and neurogenic capabilities of mesenchymal stem cells generated from bone marrow stroma have been discovered in vitro, spurring a lot of studies. Bone marrow harvesting, on the other hand, is a painful procedure for patients that only provides a minimal number of cells. BMSCs (bone marrow-derived stem cells) are the gold standard in regenerative medicine. While they are currently the gold standard for treating a range of illnesses, they have disadvantages such as a painful isolation procedure, the need for general anesthesia, and low cell yields. In contrast, ADSCs may be retrieved in large amounts during a single liposuction surgery without the need for general anesthesia. As a result, ADSC is being used to do skin flap transplantation in this research.

## 3. Methodology Used

In this section, the suggested method is explained. We have used adipose-derived stem cell (ADSC) based therapy for skin flap transplantation in skin malignant tumor resection. The schematic representation of the methodology used is represented in Figure 1.

### 3.1. Skin Flap Model and Experimental Design

All procedures involving laboratory animals were carried out in compliance with Nanjing Medical University that followed the US National Institutes of Health's Guide for the Care and Use of Laboratory Animals. The SIEA flap (6 cm × 9 cm) was grown in male Sprague–Dawley rats weighing 260 g to 320 g. Anesthesia was created and supported with a 50 mg/kg pentobarbital intraperitoneal injection, and the flaps were ischemic for 6 hours by elongating the vessel and observing blood circulation as depicted in Figure 2. Following tissue damage, the rats were arbitrarily categorized into 3 groups and given a subcutaneous administration of 100 mg of various varieties of exosomes in 200 ml of PBS or 200 ml of PBS (control) at six locations in the anterior, centre, and lateral parts of the flap to guarantee an even dispersion all through the flap.

### 3.2. Microvessel Density

The endothelial cell marker CD31 was used to evaluate the microvessel density in a flap paraffin slice (1 : 50 dilution, Abcam). The sections were then treated for 1.5 hours at room temperature with biotin-conjugated goat anti-rabbit IgG. The sections were then stained with 3,3-diaminobenzidine tetrahydrochloride (DAB) and hematoxylin counterstain. The investigators were blinded to the experimental groups when measuring the CD31-positive areas inside each skin flap segment to exclude any potential observer-dependent bias in tissue area selection.

### 3.3. IL-6 Enzyme-Linked Immunosorbent Assay (ELISA) in Cell Lysates and Conditioned Media

The ADSC (2 × 10^5^) cells were planted into 6-well plates and kept for 48 hours. After that, the supernatant and cell lysate were gathered and centrifuged. IL-6 expression was measured using ELISA kits (BioLegend, CA, USA) following the manufacturer's instructions. The absorbance of all samples was calculated at 450 nm on an EL808 microplate absorbance reader in triplicate from three different donors (BioTek, VT, USA). Standard curves made using recombinant proteins provided in the kits were used to calculate the amount of IL-6 (pg/mL).

### 3.4. Antibody Array Analysis

Following the manufacturer's directions, we used the human angiogenesis antibody array to identify angiogenic chemicals released by ADSC and Hs68 cells. The signal intensity of every point was evaluated utilizing the NIH ImageJ software and normalized to the mean of the positive control spots to assess the angiogenic particle's variability.

### 3.5. siRNA Transduction

Accell SMART pool siRNA was used to mute IL-6. A 100 M storage of siRNA was made in RNase-free water and placed at 20°C. The culture medium within every well was modified with 1 mM Sig1R siRNA or regulated nontarget Accell siRNA with a ciphered series, which had no substantial homology to human genetic sequences in Accell siRNA delivery medium after ADSCs were cultured in a 6-well plate at 70–80 percent confluence for 24 hours. Cells were cultured at 37°C for 72 hours in a 5% CO_2_ incubator. The drop in IL-6 levels was confirmed by ELISA. The si-IL-6 and si-scramble groups, derived from ADSC siRNA, were utilized to assess the significance of IL-6 in ischemia flap injury in an animal study and angiogenesis in a Matrigel-based tube formation research, accordingly.

### 3.6. Isolation of Human Adipose-Derived Stem Cells (ADSCs)

Dulbecco's modified Eagle's medium (DMEM) was combined with 10 mM HEPES and 10% foetal bovine serum to make a complete culture medium (CCM). Washing tissues and cells were performed with Hank's balanced salt solution containing 10 mM sodium HEPES, which was devoid of Ca^2+^ and Mg^2+^. Ten patients undergoing elective liposuction surgery had subcutaneous adipose tissue samples taken. The average age was 36 (24–51), the average weight was 61.4 kg, and the average BMI was 24.9 (21.5–28.3). A 3.5 mm diameter blunt cannula was used to aspirate adipose tissue from the lower abdomen. Aliquots of 10 mL washed adipose tissue were utilized in each isolation procedure. At least three distinct approaches were used to harvest cells from each patient. At 37 degrees Celsius, all cells were plated in one well of a 6-well culture plate and cultivated in 5% CO_2_. Every 2-3 days, the medium was replaced. After washing with HEPES, cells were passaged using trypsin release, counting, and seeding at suitable rates.

### 3.7. Isolation using Trypsin

ADSCs were isolated by incubation for 30 or 60 minutes at 37 C with shaking every 10 minutes and varied trypsin concentrations (025, 050, or 075, corresponding to 12.5, 25, or 37.5 g trypsin/ml of PBS with 0.2 percent EDTA, respectively). The enzyme was inactivated by adding an equal volume of the CCM and centrifuged for 10 minutes at 6009 g. The supernatant was discarded, and the pellet was treated for 5 minutes at room temperature in 10 mL red blood cell lysis buffer before centrifugation at 6009 g for 10 minutes.

### 3.8. Collagenase (COL) Isolation

Thereafter, the adipose tissue was thoroughly rinsed in PBS and digested for 30 minutes at 37 C using collagenase type I (C1 ml/ml) in the presence of 10% HEPES in the presence of moderate agitation. An equivalent amount of CCM was added to the enzyme and centrifuged at 6009 g for 10 minutes to inactivate it. This was followed by a 10-minute centrifugation at 6009 g, followed by a 5-minute incubation at room temperature with 10 ml of red blood cell lysis solution and another 10-minute centrifugation at 6009 g. The mechanical shaking of the buffer solution of the lysis of red blood cells (LBS) and the incubation with red blood cell lysis solution (NH4Cl, 10 mM NaHCO3, and 1 mM EDTA) 1:1 (v:v) for 15minutes are the two bases of this approach, which was reported by Baptista and coworkers [21]. It was centrifuged for 10 minutes at 6009 g after incubation.

### 3.9. Trypsin Isolation (T025-30, T025-60, T050-30, T050-60, and T075-30)

Different trypsin concentrations (025, 050, or 075, equivalent to 12.5, 25 or 37.5 g trypsin/ml of PBS with 0.2 percent EDTA) and incubation for 30, or 60 minutes were used to isolate ADSC at 37 C with shaking every 10 minutes. The enzyme was rendered inactive by centrifuging the suspension for ten minutes at 6009 g while adding an equivalent amount of CCM. Recentrifuged at 6009 g for 10 minutes, the pellet was incubated for 5 minutes with 10 ml red blood cell lysis solution at room temperature and discarded.

### 3.10. Centrifugation Isolation (CENT1 and CENT2)

Centrifugation at two different speeds (800 and 1,2809 g) for 15 minutes was all that was required in this procedure; no enzyme was used. Centrifugation at 6009 g for 10 minutes with 10 ml red blood cell lysis solution was performed, the supernatant was removed, and the pellet was incubated for 5 minutes at room temperature before being centrifuged again. CCM was used to resuscitate the pellets of all groups after centrifugation.

### 3.11. Determination of Population Doubling Time

From passage 3 through 12, cells were grown to 80–85 percent confluence and counted at each passage. After trypan blue staining, cell number was determined using a Neubauer chamber. The average number of days it took for cultures generated from at least three different donors to double their population was calculated. The population doubling time for the various cultures was estimated using the formula:

(1) $$\begin{array}{c} \text{population doubling time}=\log\left(\text{final cell number}\right)-\log\left(\text{starting cell number}\right)=K9T, \end{array}$$

where *K* is the generation constant and *T* is the time in days.

### 3.12. Immunophenotyping

Flow cytometry was used to examine the surface markers of the separated ADSCs. Trypsin dissociated the cells, which were then centrifuged and treated with phycoerythrin (PE)- or fluorescein isothiocyanate (FITC)-conjugated antibodies specific for human CD90.2, CD45, CD34, CD44, CD73, CD117, and CD11b for 30 minutes at 4 C. The cells were examined using the CellQuest software and a FACSCalibur flow cytometer with a 488 nm argon laser. A total of 10,000 events were gathered.

### 3.13. Differentiation of Isolated ADSCs

Isolated ADSCs were differentiated by culturing cells between passages 4 and 7 at 2.2 × 9 × 10^5^ cells/cm^2^ in specialized media for 4 weeks, with the medium changed every 3 days. CCM was supplemented with 10^−8^ M dexamethasone, 5 mg ascorbic acid 2-phosphate ml^−1^, and 10 mM b-glycerophosphate for osteogenic differentiation. Washing once with PBS, fixing with 4 percent paraformaldehyde in PBS for 15–30 minutes at room temperature, and staining with Alizarin Red S indicated calcium buildup in differentiated cells. ADSCs were grown in the CCM supplemented with 10^−8^ M dexamethasone, 2.5 mg insulin ml^−1^, 100 mM indomethacin, and 3.5 mM rosiglitazone for adipogenic development. Adipocytes were stained with Oil Red O solution for 5 minutes at room temperature after being fixed with 4 percent paraformaldehyde in PBS for 1 hour at room temperature. The following methods for isolation of ASCs were tested.

### 3.14. Statistical Analysis

There were three to six different studies that yielded the mean SEM and were reported as a fold change in comparison to the control value. We used a one-way ANOVA and Fisher's exact test for all of our statistical evaluations. For each of the 12 studies, a *P* value of 0.05 significance level was required.

## 4. Results and Discussion

This section explains the performance analysis of the suggested methodology. All of the methods evaluated in this study yielded viable cells.

As of from Figure 3, IL-6 neutralising antibody (anti-IL-6), siRNA for IL-6 transfection (si-IL-6), and transfection of a scrambled oligonucleotide sequence (control) were used to collect the conditioned medium from ADSCs (si-Scramble). Immunofluorescent labelling was used to assess IL-6 expression in I/R skin flaps with or without CM, IgG, anti-IL-6, si-Scramble, or si-IL-6 therapy. IL-6 (arrow) expression was significantly higher in CM-, IgG- and si-Scramble-treated I/R flaps than that in I/R alone or immunosuppressive treatments.

The histological grading method was used to assess the healing of the skin flap. The quantity of inflammation, collagen deposition, epithelialization, and hair follicles was among the histological findings. Each parameter was evaluated on its own and received a score of 0–3. After the five-day postoperative care of the i/r mice with skin flap transplantation, the total score is zero based on the four metrics (Figure 4). In the examination of viability in tissues produced from different isolating techniques, the percentage of cell viability was higher in 2 categories employing trypsin (T025-30 and T025-60) comparable to collagenase (*p* < 0.05) (Figure 3). The T025-30 showed a higher proportion of cell viability than the LBS category (*p* < 0.05). None of the trypsin techniques indicated a significant difference.

Figure 5 depicts the number of isolated cells. The traditional collagenase-based ADSC isolation approach yielded considerably more cells than the other protocols (*p* < 0.001). The lack of statistically significant variations in cell production between all trypsin groups and LBS was likely owing to the large standard deviation resulting from patient variances.

The population doubling duration was identical in all cultures (Figures 6 and 7) and stayed unchanged. The population doubling time in bone marrow MSCs increased considerably whereas ADSCs from the same patient remained steady, indicating that such cells are probably more suited for protracted proliferation in vitro.  Figure 8 illustrates the flap survival rate in percentages for both bone marrow stem cells and adipose-derived stem cells. The graph clearly shows that ADSC has the highest survival rate.

## 5. Conclusion

Given that the trypsin protocol for ADSC isolation is 40 times cheaper than collagenase, has a 5-fold lower yield, and produces cultures with similar average proliferation capacity, we believe that trypsin is an important alternative protocol to the traditional method for isolating adipose-derived stem cells. Our findings suggest that incubation with trypsin at a lower dosage (25 percent) for 60 minutes is the optimal strategy for replacing collagenase tissue digestion. Furthermore, based on the differentiation outcomes, we believe that this isolation approach could be a potential method for bone tissue engineering research. We also looked into how exosomes released by ADSC affected flap survival during tumor excision. The key discovery was that ADSC increased neovascularization in the skin flap after transplantation and reduced inflammatory responses and apoptosis. These findings show that using ADSCs as a pretreatment for exosome-based skin flap survival could be beneficial.

## Figures and Tables

**Figure 1:** Schematic representation of the methodology used.

**Figure 2:** Experimental design.

**Figure 3:** Expression of IL-6.

**Figure 4:** Skin flap recovery system.

**Figure 5:** Cell yield of viable cells (×104).

**Figure 6:** Cell viability of viable cells (%).

**Figure 7:** Cell population doubling time.

**Figure 8:** Comparison of flap survival rate (%) for BMSC and ADSC.

## Data Availability

All data included in this study are available upon request by contacting the corresponding author.
